# The Impact of Catchment Land Use Land Cover Changes on Lake Dandi, Ethiopia

**DOI:** 10.1155/2022/4936289

**Published:** 2022-06-17

**Authors:** Mulugeta B. Dega, Alemayehu N. Emana, Habtamu A. Feda

**Affiliations:** ^1^College of Natural and Computational Sciences, Ambo University, Ambo, Ethiopia; ^2^Geomatics Engineering, Ambo University, Ambo, Ethiopia

## Abstract

Highland freshwater lakes are currently threatened with catchment land use land cover changes particularly in developing countries like Ethiopia despite their wide range of valuable ecosystem services. This study was conducted to assess trends of catchment land use land cover change and associated impacts on a highland Lake, Dandi over three decades from 1990 to 2020 years period based on GIS (ArcMap 10.4.1) and remote sensing (ERDAS Imagine 14) software as well as questioner survey, key informant interviews, and field observation. The study covered 3,794 ha with five major land use land covers, namely mixed agriculture/settlement, bush-/shrubland, grassland, bare land, and water body (Lake Dandi). The assessment revealed that farmland/residential area increased by 593 ha (35.34%), while bare land, grassland, shrubland, and Lake Dandi decreased by 290 ha (26.12%), 218 ha (12.15%), 57 ha (6.85%), and 28 ha (19.53%), respectively. Responses also indicated increased farmland/settlement area (66.66%) and declined areas of bare land (84.63%), bush-/shrubland (84.86%), grassland (96.96%), and Lake Dandi (61.05%). Furthermore, responses indicated expanding agricultural land use (48%), population growth (38%), climate change (32%), overgrazing (30%), and poverty (28%) as major factors currently threatening the lake and its ecosystem services. Field observation also revealed expansion of agricultural land use in the catchment of Lake Dandi including in steeper slopes and hillsides that might exacerbate on-site soil erosion as well as lake sedimentation and toxic contamination. Thus, results indicated deterioration in the storage capacity and water quality of Lake Dandi due to catchment land use land cover change that might in turn adversely affect its ecosystem services and the resident biota suggesting urgent intervention.

## 1. Introduction

All over the world, lakes are hotspots of biodiversity and provide various ecosystem services such as water quality maintenance, carbon sequestration, shoreline protection, and recreational values [1]. Although lakes cover only a small part of the Earth, they contribute 40% of the annual global ecosystem services [2]. Natural and man-made lakes together store more than 90% of the world's surface freshwater resources and are heavily used for a variety of human activities, including drinking, fishing, irrigation, navigation, and recreation [3]. Freshwater is an essential natural resource for humankind and central to sustainable development as well as poverty alleviation.

Well-managed lakes are among the most productive ecosystems and provide the opportunity for sustainable development, helping to meet the needs for improved living standards in developing countries such as Ethiopia [4]. Nevertheless, related to a lack of the necessary awareness and poverty, human activities have severely degraded the ecosystems largely in developing countries, diminishing their ability to provide valuable ecosystem services and driving species to extinction, which is a matter of great concern. Though there is a growing recognition of the need for their conservation, lakes continue to be lost throughout the world [5], and half of the world's lakes have been lost in the twentieth century [6]. With their rich, seasonally inundated soils, lakes have become “new agricultural frontiers” that provide important farming resources for a wide range of sectors [7]. That is the main reason why lake degradation and loss are likely to aggravate the socioeconomic pressures on the rural poor of the developing nations while reducing the options available for maintenance of environmental quality as the main consequence [8]. Poor lake water quality also adversely affects human health, economic health, and ecosystem health that are interrelated [9].

Ethiopia, with its different geological formations and climatic conditions, is endowed with over 15 natural lakes including Lake Dandi and many man-made reservoirs that constitute a valuable natural resource storing freshwater for domestic consumption, irrigation, and some industrial purposes, generating electricity, recreation, domestic animals, and supporting many species of harvestable fish and birds of great tourism attraction. However, some of these lakes are currently undergoing degradation both in quantity (e.g., Lake Abijata, Lake Haromaya, and Lake Chamo) and quality (e.g., Koka Reservoir and Lake Ziway) due to human activities, and Lake Dandi is not an exception. This study was conducted to assess the impacts of catchment land use land cover change on Lake Dandi.

## 2. Materials and Methods

### 2.1. Description of the Study Area

The study was conducted on number “8” shaped central highland natural freshwater Lake Dandi and its catchment that covers 820 ha and is located between 8°43′N–9°17′N and 37°47′E–38°20′E (Figure 1), about 108 Km, 60 Km, and 31 Km away from the capital (Addis Ababa), zonal town (Ambo), and district town (Ginchi), respectively [10]. Lake Dandi is the source of the Huluka River that constitutes the main source of water supply for Ambo town and its surroundings. Dandi District has a tropical climate with mean minimum and maximum temperatures of 9.6 C and 23.3 C, respectively [11]. The district has a total area of 79,939.29 ha lying at an average altitude between 2,000 ma.s.l and 3,288 ma.s.l and is divided into high land (29%) and moderate (71%) [12]. The annual average rainfall of the district is 900–1,400 mm, and rainfall of the area is bimodal, with unpredictable short rains from March to April and the main season ranging between June and September. The erratic nature of the rainfall in the area made farming unpredictable and generally put it at a low level of productivity [11]. Dandi district has 38 rural kebeles (local administrative units) and seven urban and semiurban out of which three towns, namely Ginchi, Asgori, and Boda, have municipal status [13]. The total population of the district is 167,132 with 84,476 males and 82,656 females [12].

The economic activities of the majority of the population of the district are characterized by mixed farming. The dominant economic activity in the Dandi district is agriculture that dominantly relies upon seasonal rainfall, while cash crops such as potatoes on the high land use small irrigations. The major crops grown in the district are teff, wheat, sorghum, and barley. Domesticated animals are also found in the district with a greater proportion comprising about 801,444 sheep, 160,641 cattle, 17,729 goats, 87,235 poultry, 21,744 horses, 2,199 mule, and 21,395 donkeys that serve as the major sources of income for the local community [11]. The natural vegetation in the study area was under heavy pressure related to the growing population, expansion of agricultural lands, fuel wood collection, and charcoal production for market [14].

The agricultural practices are traditional and unsustainable adversely affecting the balance of the relationship between people, land, and their livelihoods patterns. The effect of this imbalance was manifested in the occurrence of unsustainable agricultural and natural resource management practices. These include cultivation of hillsides and steep slopes, deforestation of natural vegetation (forest and shrubs), diminishing of indigenous trees and wild animals, degradation and shrinkage of grazing areas, farming practices that facilitate soil and nutrient erosion, less water infiltration, and gully formations, which deteriorates land productivity.

### 2.2. Satellite Images

The impact of catchment land use land cover change on Lake Dandi was assessed from 1990 to 2020 based on LULC data of the study area obtained from time series of satellite images using remote sensing (multitemporal and differential resolution remote sensing data, which includes Landsat Thematic Mapper, Enhanced Thematic Mapper, and Operational Land Imager—TM, ETM, and OLI—images) from the United States Geological Survey (USGS).

Preprocessing of satellite images before detection of changes is a vital procedure and has the unique aim of building a more direct association between the biophysical phenomena on the ground and the acquired data [15]. Data were preprocessed in ERDAS Imagine for georeferencing and subsetting of the image on the basis of area of interest (AOI). Standard image processing techniques such as image extraction, rectification, restoration, atmospheric and sun angle correction, and radiometric correction and classification were used for the analysis of satellite imageries using ERDAS Imagine and impact tool software. Landsat imageries of three bands [11, 12, 15] for Landsat TM, whereas bands [11–13] to Landsat-8 were used in image enhancement to identify changes in land use/land cover features. All satellite images had an original format in TIFF. They were exported to image format in ERDAS Imagine 2015 software using the layer stack function. The images were georeferenced into the same map projection of WGS (World Geodetic System) 1984 Zone 37N.

All satellite images were subset for covering only the study area using the shape file of the study area. In order to interpret and discriminate surface features clearly, all satellite images were composed using red green blue (RGB) color composition. False color composites (FCC) of satellite imageries were prepared for the years 1990, 2000, 2010, and 2020 using band 4 (NIR), band 3 (Red), and band 2 (Green) combinations.

Image classification is necessary to convert image data to thematic data. According to Lilles and Kiefer [16], the overall objective of image classification procedures is to automatically categorize all pixels in an image into land use and land cover classes. As there was no prior knowledge about the study area, an unsupervised classification method was used to get an idea of the approximate land use and land cover of the study area and to use it in sampling prior to the field visit. This technique was used for classifying features in an image, which have common characteristics into clusters based on the software analysis of an image without the user providing sample classes [17]. The maximum number of clusters, maximum cluster size, and minimum distance were defined for computer uses to locate arbitrary vectors as the center points of the clusters. Then, each pixel was assigned to a cluster using the minimum distance cluster centroid decision rule. The result from this process was a raster map, each pixel having a class of the cluster.

A supervised classification was performed using the maximum likelihood algorithm methodology for the extraction of land use and land covers of the study area in ERDAS Imagine software. Five land use and land covers such as agriculture/settlement, grassland, bare land, shrub-/bushland, and lake or water body were considered as training areas in image classification based on samples collected from fields. These major land-use and land-cover types were identified by using the field data and satellite images of Landsat TM, 1998, ETM, 2008, and OLI, 2018. In ERDAS Imagine software, the signature editor was created for defining classes. By using area of interest (AOI) tools with the help of Google Earth Pro, the boundaries and number of pixels for each class were added to the signature editor.

Next, the decision-making phase was taken place, and the maximum likelihood algorithm was selected because of the advantage of considering the center of the clusters together with shape, size, and orientation. It was difficult to identify settlements especially rural settlements from agricultural land on a 30 m spatial resolution image, and in most cases, the two are spatially integrated. Therefore, settlements were grouped under agricultural land covers. Finally, land use and land cover maps for the years 1990, 2000, 2010, and 2020 were classified. The land use land cover types and description of the study area are summarized in Table 1.

The common way to represent classification accuracy was taken in the form of an error matrix. An error matrix is a square array of rows and columns and presents the relationship between the classes in the classified and reference data. Reference data used for accuracy assessment were obtained from field observations. Using the ERDAS Imagine software accuracy assessment utility, reference random test pixels in the study area were located, which were not used in the training of the classification algorithm to eliminate the possibility of bias of training samples chosen in classification.

A set of reference pixels representing geographic points on the classified image is required for the accuracy assessment. These points were verified and labeled against the reference data. Error matrices were then designed to assess the quality of the classification accuracy of 1990, 2000, 2010, and 2020 LULC maps. Overall accuracy was computed by dividing the total correct number of pixels (i.e., summation of the diagonal) by the total number of pixels in the matrix (grand total). Various standard threshold levels were applied to the lower and higher tail of each distribution in order to find the threshold value that produced the highest change classification accuracy [18]. Producer's accuracy refers to the probability of a reference pixel being classified correctly. It is also known as omission error because it only gives the proportion of the correctly classified pixels.

It was obtained by dividing the number of correctly classified pixels in the category by the total number of pixels of the category in the reference data. User's accuracy assesses the probability that the pixels in the classified map or image represent that class on the ground [19] and is obtained by dividing the total number of correctly classified pixels in the category by the total number of pixels on the classified image. Kappa coefficient was also used to assess the classification accuracy. It expresses the proportionate reduction in error generated by a classification process compared with the error of a completely random classification [19].

LULCC were computed as follows:

(1) $$\begin{array}{c} \text{Total LULCC}=\text{Area of final year}-\text{Area of initial year,} \end{array}$$

(2) $$\begin{array}{c} \text{Percentage LULCC}=\left(\frac{\text{Area of finl year}-\text{Area of initial year}}{\text{Area of initial year}}\right)\;\;\times 100, \end{array}$$

where Area is the extent of each LULC type. The positive values suggest an increase whereas negative values imply a decrease in extent.

### 2.3. Local Community Perception

Local community perception of the land use land cover changes and their impacts on Lake Dandi were assessed based on households' using structured questionnaires survey and key informants interviews. The survey involved 176 sample household heads selected from the target population of 300 heads who lived in the surrounding two rural kebeles (Dandi Mumicha and Dandi Sulu) for more than 30 years (Table 2).

The sample size was determined following Yamane [20], and respondents were selected using a simple random sampling technique.

(3) $$\begin{array}{c} n=\frac{N}{1+N\left(e^{2}\right)}, \end{array}$$

where *n* = is the sample size, *N* = is the study population, and *e* = was the level of precision.

By using formula (3), sample size was calculated as follows:

(4) $$\begin{array}{c} n=\frac{300}{1+300\left(0.05^{2}\right)}, \end{array}$$

where *n* = 176.

(5) $$\begin{array}{c} n1=\frac{n^{*}\times n}{N}=\frac{100\times 172}{300}=58, \end{array}$$

(6) $$\begin{array}{c} n2=\frac{n^{*}\times n}{N}=\frac{200\times 172}{300}=118, \end{array}$$

where *n*^*∗*^is the proportional sample from each kebele, *n* is the sample size for the study, and *N* is the study population.

Key informant interview was conducted with a total of eight informants identified (five from each Kebele and three from the district level; Table 3). Four farmers and four community elders who lived in the area for more than 30 years and two agricultural developments agents (DAs) were involved in the interview from the two kebeles. At the district level one expert, one head from the district Environment, Forest and Climate Change Authority (EFCCA) as representative of political leader, and one expert from the Culture and Tourism Office were involved as key informants. Semistructured checklists were designed to administer the key informant interviews (KIIs).

Furthermore, field observation was made to verify the information obtained through other data collection tools and assess the overall topographic conditions, socioeconomic characteristics, grazing patterns, and status of the lake ecosystem. The observation also covered soil and water conservation practices, livestock, grazing land, the status of infrastructure, as well as the scientific and traditional maintenance of degraded land.

## 3. Results

### 3.1. Land Use and Land Cover Analysis

The satellite imagery data revealed five major LULC types including agricultural/settlement land, bush-/shrubland, grassland, bare land, and Lake Dandi that together accounted for about 3,794 ha (Figure 2). The satellite images further detected decline in bare land, bush-/shrubland, grassland, and Lake Dandi whereas increase in the farmland during the study period (Figures 2 and 3).

The satellite data for 1990 revealed 1,281 ha (33.76%) bare land, 769 ha (20.27%) lake area, 748 ha (19.71%) agricultural/residential land, 679 ha (17.89%) grassland, and 317 ha (8.35%) bush-/shrubland. On the other hand, data imagery of the year 2020 indicated 1,341 ha (35.34%) agricultural/residential land, 991 ha (26.12%) bare land, 741 ha (19.53%) lake area, 461 ha (12.15%) grassland, and 260 ha (6.85%) bush-/shrubland.

### 3.2. Accuracy Assessment

Accuracy assessment is a general term used to compare the classification to geographical data that are assumed to be true, in order to determine the accuracy of the classification process. The common way to represent classification accuracy was taken in the form of an error matrix. An error matrix is a square array of rows and columns and presents the relationship between the classes in the classified and reference data. Reference data used for accuracy assessment were obtained from field observations. A set of reference points were taken to assess its accuracy. Accuracy assessment points were independent of those used in land-cover class assignments. Using the ERDAS Imagine software accuracy assessment utility, reference random test pixels in the study area were located, which were not used in the training of the classification algorithm to eliminate the possibility of bias of training samples chosen in classification. A set of reference pixels representing geographic points on the classified image is required for the accuracy assessment. These points were verified and labeled against the reference data. Error matrices were then designed to assess the quality of the classification accuracy of 1990, 2000, 2010, and 2020 LULC maps. Overall accuracy was computed by dividing the total correct number of pixels (i.e., summation of the diagonal) by the total number of pixels in the matrix (grand total; Tables 4–7). Various standard threshold levels were applied to the lower and higher tail of each distribution in order to find the threshold value that produced the highest change classification accuracy [18]. Producer's accuracy refers to the probability of a reference pixel being classified correctly. It is also known as omission error because it only gives the proportion of the correctly classified pixels. It is obtained by dividing the number of correctly classified pixels in the category by the total number of pixels of the category in the reference data. User's accuracy assesses the probability that the pixels in the classified map or image represent that class on the ground [19] and is obtained by dividing the total number of correctly classified pixels in the category by the total number of pixels on the classified image. Kappa coefficient was also used to assess the classification accuracy. It expresses the proportionate reduction in error generated by a classification process compared with the error of a completely random classification [19]. Kappa statistic incorporates the off-diagonal elements of the error matrices (i.e., classification errors) and represents agreement obtained after removing the proportion of agreement that could be expected to occur by chance. The ground truth data (GPS Point) were utilized in the classification report as the independent data set from which the classification accuracy was compared for the current year (2020). For the other maps mean for 1990, 2000, and 2010, the reference points were collected from Goggle Earth with the highest resolution and used to validate the accuracy of the classified image.

The kappa coefficient lies typically on a scale between 0 and 1, where the latter indicates complete agreement and is often multiplied by 100 to give a percentage measure of classification accuracy. In this study, kappa coefficient of the four periods 1990, 2000, 2010, and 2020 was found to be 0.65, 0.74, 0.80, and 0.85, respectively (Tables 4–7). The overall accuracy of the 1990, 2000, 2010, and 2020 years was 83.78%, 84.14%, 84.48%, and 86.20%, respectively. Therefore, this finding shows that there is a strong agreement between the classification map and the ground reference information indicating kappa coefficient ranges of all the LULCC classes were excellent.

### 3.3. Change Detection on Land Use Land Cover of the Study Area

The satellite image data of the study area revealed that agricultural land/settlement increased while other classes declined throughout the study periods. Over the three decades, that is, 1990–2020, agricultural land/settlement increased by 593 ha (35.34%) with an average change rate of 79.27 ha/year. On the other hand, bare land showed the highest decrease, that is, 390 ha (26.12%) with an average change rate of 28.24 ha/year (Table 8). Grassland revealed a low change of 218 ha (12.15%) and reduced by 30.10 ha/yr. Bush-/shrubland decreased by 57 ha (6.85%) with 17.98 ha/year, whereas Lake Dandi declined by 28 ha (3.64%) with about 10 ha/year.

### 3.4. Demographic Characteristics of Respondents

All the respondents were older than 30 years (Table 9) that implies that the respondents had adequate exposure to trends of catchment land use land cover change and its impacts on Lake Dandi during the study period. The majority of the respondents were married males and illiterate/lower educational status.

Out of the 176 respondents, 118 (66.66%) confirmed the expansion in agricultural land use, and 171 (96.96%) replied that grassland has been converted to farmland (Table 10) resulting in overgrazing (Table 11). Furthermore, 150 (84.86%) and 61 (34.84%) of the respondents indicated a decline in the areas of bushland and Lake Dandi, respectively, during the past three decades.

Among other things, the responses indicated expansion of agricultural land use (48, 27.28%), population growth (38, 21.59%), and climate change (32, 18.18%) as the major factors currently threatening Lake Dandi and its ecosystem services (Table 8).

## 4. Discussion

Satellite images detected changes in all the land use land cover types in the study area during 1990–2020. The result indicated an increased agricultural/settlement land use most probably at the expense of the rest of land use land covers, namely grassland, bush-/shrubland, bare land, and water body (Lake Dandi). The findings of this study revealed a strong agreement between the classification map and the ground reference information indicating that the kappa coefficient ranges of all the LULCC classes were excellent. This is in agreement with Tamiru Lemi [21] who reported a decrease in the area of Ethiopian rift valley lakes, namely Abiyata, Ziway, Langano, and Shalla lakes, from 1985 to 2015. Most of the studies conducted [22, 23] also indicated that agriculture is the primary cause of the LULC dynamics in the central highland of Ethiopia and in line with the present finding.

Results further revealed that Lake Dandi was being encroached over time by catchment land degradation related to population growth and attendant vegetation removal, expanding farmland, cultivating hillsides, overgrazing, sedimentation due to soil erosion, and conversion of the lake into other land use types, which is in agreement with Tamiru Lemi [21]. Land use land cover change in the catchment of Lake Dandi might adversely affect the storage capacity and water quality of the lake and consequently its ecosystem services. This may degrade both the quantity and quality Huluka River (the outflowing river) water and adversely affect downstream users including zonal town residents and the surroundings for various purposes especially during the rainy season if not given due attention. Furthermore, it may undermine its huge potential for cultural services, which are currently under development.

About 27.28% of the respondents indicated a decline in farmland that might be partly attributed to the illiterate/low educational level and old age of some sample respondents included to get the necessary information on the point in focus over the 30 years period. According to the respondents, productivity declined despite the expansion in agricultural land use that might be because of land degradation. LULC changes are dynamic and nonlinear, that is, the conversion from one land use to the other does not follow a similar pattern, due to natural or anthropogenic factors such as policy change, population growth, and a decrease in the productivity of land [24]. Land use policy in Ethiopia has been changed remarkably since 1972 because there was a change of regime from feudal to the Dergueregime. Haile Selassie regime encouraged commercialization and mechanization of agriculture and firms were easily accessing tractors and fertilizers on a loan basis. However, during the Military Dergueregime, land became a communal property (land reform) with the promotion of cooperatives in the villagization program across the country that resulted in depletion of natural resources including lakes, increased cultivated land, increased forest clearance, and high level of land degradation. The Ethiopian People Revolutionary Democratic Front (EPRDF) sustained the same land policy that encouraged smallholders to put extra forest area into cultivation to produce high-value crops for possible markets and agro-processing plants favoring a mixed economy [25].

The respondents suggested integrated watershed management involving terracing, tree planting, sustainable agricultural practices, and controlled grazing as a way forward to sustain the lake and its vital ecosystem services. Furthermore, they emphasized the relevance of poverty reduction, diversifying livelihoods, effective land-use policy, tenure security, coordination, and institutional collaboration and accountability to ensure sustainable development of the ecosystem.

## 5. Conclusions and Recommendations

Predominantly continued expansion of agricultural land use in the steeper topography catchment might have degraded the landscape and caused a decline in the area of Lake Dandi. This may threaten the biodiversity of the lake and adversely affect its ecosystem services including water supply to Ambo town and its surrounding through Huluka River as well as its ecotourism potential. The ongoing effort to develop the ecotourism potential of Lake Dandi should be encouraged as this could at the same time ensure its ecosystem services besides the intended direct economic benefits. Developing the ecotourism potential of the lake on a sustainable basis requires integrated watershed management and proper monitoring to avoid possible contaminations and protect downstream users.

## Figures and Tables

**Figure 1:** Map of the study area.

**Figure 2:** Map of LULC of the study area from 1990 to 2020.

**Figure 3:** Trends in LULC.

**Table 1:** Land use land cover type and the corresponding description.

LULC types	Description
Bare land	Land area with no dominant vegetation cover on at least 90%.

Bush-/shrubland	Land area covered by alpine vegetation communities dominated by low, woody, self-supporting, multistemmed plants branching at or near the ground, between 0.2 and 2 m in height.

Agricultural/settlement	Made to include areas allotted to rain-fed cereal crops (e.g., legumes, barley, teff, and wheat) and horticultural crops particularly vegetables (e.g., onion, potato, and cabbage). Crop cultivation, both annuals and perennials, mostly in subsistence farming and the land covered by rural villages and scattered rural settlements surrounded by Enset.

Grassland	Both communal and/or private grazing lands that are used for livestock grazing. The land is basically covered by small grasses, grass-like plants, and herbaceous species. It also includes land covered with a mixture of small grasses, grass-like plants, and shrubs less than 0.2 m, and it is used for grazing.

Lake	Land area covered by water.

Source: Field survey 2021.

**Table 2:** Sample size.

Kebele	Total population	Sample size
Dandi Mumicha	200	118
Dandi Sulu	100	58
Total	300	176

**Table 3:** Key informants interview.

Key informants	Administrative unit	Number
Elders (age >50 years)	Kebele	4
Farmers	Kebele	4
DA (development agent)	Kebele	2
Culture and tourism expert	District	1
Environmental expert	District	1
Environmental leader	District	1
Total		13

**Table 4:** Accuracy assessment for supervised classification of Landsat TM 1990.

	Reference data							
Classified data	LULC	FL/S	Bare	GL	BL	Lake	Total	**UA%**
	FL/S	**47**	2	4	4	0	**57**	**76.19**
	Bare	1	**38**	3	3	1	**46**	**74.19**
	GL	2	2	**33**	0	2	**39**	**75**
	BL	0	1	4	**37**	1	**43**	**78.57**
	Lake	2	1	2	1	**31**	**37**	**72.72**
	Total	**52**	**44**	**46**	**45**	**35**	**222**	
	**PA%**	**90.38**	**86.36**	**71.73**	**82ct.22**	88.57		

Over all accuracy = 47 + 38+33 + 37+31/222 = 83.78% and overall kappa statistics = 0.65.

**Table 5:** Accuracy assessment for supervised classification of Landsat TM 2000.

	Reference data							
Classified data	LULC	FL/S	Bare	GL	BL	Lake	Total	**UA%**
	FL/S	**48**	1	4	4	1	**58**	**82.75**
	Bare	1	**39**	3	3	1	**47**	**82.97**
	GL	2	2	**34**	0	2	**40**	**85.00**
	BL	0	2	4	**38**	0	**44**	**86.36**
	Lake	2	1	2	1	**32**	**38**	**84.21**
	Total	**53**	**45**	**47**	**46**	**36**	**227**	
	**PA%**	**90.56**	**86.66**	**72.34**	**82.60**	88.88		

Over all accuracy = 48 + 39+34 + 38+32/227 = 84.14% and overall kappa statistics = 0.71.

**Table 6:** Accuracy assessment for supervised classification of Landsat TM 2010.

	Reference data							
Classified data	LULC	FL/S	Bare	GL	BL	Lake	Total	**UA%**
	FL/S	**49**	2	4	4	0	**59**	**83.05**
	Bare	1	**40**	3	3	1	**49**	**81.63**
	GL	2	2	**35**	0	2	**41**	**85.36**
	BL	0	1	4	**39**	1	**45**	**86.66**
	Lake	2	1	2	1	**33**	**39**	**84.61**
	Total	**54**	**46**	**48**	**47**	**37**	**232**	
	**PA%**	**90.74**	**86.95**	**72.91**	**82.97**	89.18		

Over all accuracy = 49 + 40+35 + 39+33/232 = 84.48% and overall kappa statistics = 0.80.

**Table 7:** Accuracy assessment for supervised classification of Landsat TM 2020.

	Reference data							
Classified data	LULC	FL/S	Bare	GL	BL	Lake	Total	**UA%**
	FL/S	**50**	0	4	4	0	**58**	**86.20**
	Bare	1	**41**	3	3	1	**49**	**83.67**
	GL	0	2	**36**	0	2	**40**	**90.00**
	BL	0	1	4	**40**	1	**46**	**86.69**
	Lake	2	1	2	1	**33**	**39**	**84.61**
	Total	**53**	**45**	**49**	**48**	**37**	**232**	
	**PA%**	**94.33**	**91.11**	**73.46**	**83.33**	89.18		

Overall accuracy = 50 + 41+36 + 40+33/232 = 86.20% and overall kappa statistics = 0.85. *Note.* FL/*S* = farmland/settlement, GL = grassland, BL= bushland, PA = producer accuracy, and UA = user accuracy.

**Table 8:** Land use land cover area change during 1990–2020.

LULC class	1990–2000		2000–2010		2010–2020		1990–2020	
	ha/year	%	ha/year	%	ha/year	%	ha/year	%
Bare land	−241	−17.45	−68	−5.96	−81	−7.55	−390	−28.24
Bushland	−29	−9.14	−8	−2.77	−20	−7.14	−57	−17.98
Farmland	227	30.34	165	16.92	201	17.63	593	79.27
Grassland	−47	−6.92	−80	−12.65	−91	−16.48	−218	−32.10
Lake	−10	−1.31	−10	−1.31	−8	−1.06	−28	−3.64

**Table 9:** Characteristics of the respondents.

Attribute	Frequency	Percentage (%)
Age		
30–50	80	45.45
51–70	51	28.97
>70	45	25.56

Educational status		
Illiterate	96	54.54
1–8	35	19.9
9–12	26	14.77
Above grade 12	19	10.8

Total	176	100

Sex		
Male	121	68.75
Female	55	31.25

Marital status		
Single	15	8.52
Married	137	77.84
Divorced	11	6.25
Widowed	13	7.4

Total	176	100

**Table 10:** Responses on LULCC in the study area over the study period.

LULC class	Households responses					
	Increase	%	Decrease	%	No change	%
Bare land	—	—	147	84.63	29	15.15
Bush-/shrubland	10	5.3	150	84.86	16	9.84
Farmland/settlement	118	66.66	48	27.28	10	6.06
Grassland	5	3.04	171	96.96	—	—
Lake	61	34.84	95	61.45	20	3.78

**Table 11:** Responses on factors threatening Lake Dandi.

Threat	Frequency	Percentage (%)
Population growth	38	21.59
Agricultural expansion	48	27.28
Overgrazing	30	17.04
Poverty	28	15.90
Climate change	32	18.18
Total	176	100

## Data Availability

The necessary data have been included in the article.
